# Cognitive Attitudes of International Mainstream Media to China during the Contaminated Water and Human Health Under Big Data

**DOI:** 10.1155/2022/9033781

**Published:** 2022-09-12

**Authors:** Kaixi Ji, Zitong Yang, Mengqian Zhou

**Affiliations:** School of Liberal Arts, Nantong University, Nantong 226000, China

## Abstract

The water pollution affecting human health is a crisis and big test, which tests the mainstream news media's ability and level of communication to respond to major public opinions and public emergencies. The contaminated water is a crisis and a major test, which tests the ability and level of communication of major news outlets to respond to important common views and emergencies. It aims to understand the perception and attitude of the international mainstream media towards China during the contaminated water. The work sorted out the mainstream media's reporting of China from the contaminated water to the present and selected the New York Times, The Times, and the Guardian as examples. We could understand the changes in China's international image during the water pollution through these mainstream media reports on China. The results show that these media reports on water pollution in China mainly focused on negative public opinion, which accounted for more than 70% of the total number of reports. Western developed countries such as the United Kingdom and the United States are out of consideration for their national interests. Using mainstream media to create public opinion that is not conducive to China, advocating “neo-colonialism”, “China threat theory” and other false statements, trying to limit China's influence, due to the difference in cognitive habits and the influence of British and American media hegemony also affects the country The communication and understanding between the two have brought obstacles.

## 1. Introduction

The stage of international politics presents an important feature of “political mediation” in the context of the “media society” era. International news and media coverage in various countries is important political information, which profoundly influences the trend of international politics [1]. As an interdisciplinary research field, political communication provides a good perspective for studying the spread of international hot events. The complex political environment and media environment put forward higher requirements for countries to formulate and implement political communication strategies [2].

With the growing rise of China, the issue of China's national image abroad has increasingly become a research hotspot in Chinese academic circles, especially in international relations and communication [3]. An important source of China's image is the recognition of Chinese groups overseas, especially as Chinese tourists have gone abroad on a large scale in recent years. The recognition of Chinese tourists by overseas people, especially through the local mainstream media, is the recognition of Chinese tourists and has become an important source of overseas Chinese image. It has been nearly two years since the outbreak of the new crown epidemic.

At present, the water pollution situation in China is basically under control and the economic recovery is in good shape. However, the water pollution situation is out of control and there are endless rumors that water pollution is spreading from China. Chinese media continue to refute rumors, but the effect is not obvious due to factors such as the Chinese media's right to speak in the world [4].

The work combed through the international mainstream media's perception and attitude towards China during the water pollution, systematically analyzes reports and reader comments through qualitative, quantitative analysis, comparative analysis, case studies and other comprehensive research methods, presenting and revealing the international mainstream The political communication practice landscape of news media and the hidden influencing factors behind it analyzes and explores the perception of China by mainstream international media.

Experts have studied the influence of media propaganda on the country's image. Chen proposed the “secondary communication method” and “selective attention and understanding” of information. Lazarsfeld summarized the “Five W” communication modes and environmental testing, social coordination, and understanding in the “Structure and Function of Social Communication”. Three basic social functions of cultural heritage [5]. Goldman DT studied the decision-making process of the political system and determined many indicators to measure the adaptability of the political system [6]. The input-output system model proposed by Tatar A puts forward the role of the “five levels of waterfall model” information flow in national decision-making [7]. Yousef MS combined the results of international political communication with international events in his research International Political Communication: Control and Influence [8]. Popova A Y wrote International Image Communication. The research highlights the role of international political communication, but overall, it is relatively scattered and not clear enough [9]. Setiyo M started with the constructive interaction of constructivism, especially the constructive role of ideas when analyzing and exposing the source of negative reports. Material analysis and data comparison are used to understand the theoretical origin and nature of the problems related to negative media reports in China. It is a pioneering work in China, but there are still some drawbacks in material selection and theoretical argumentation [10].

The novelty of the work lies in the research of this article. In this article finds that the light of their own national interests, developed countries such as the United Kingdom and the United States use the media to create public opinion that is unfavorable to China, supporting the “new colonialism”, “Chinese threat theory”, etc. Untrue remarks try to limit China's influence. Meanwhile, the difference in cognitive habits and the influence of the hegemony of the British and American media have also brought obstacles to cognition and communication between countries. The mainstream British and American media represented by the “New York Times”, “The Times” and “The Guardian” have always adopted western values as the standard and hope to include China in their dominant international system; China's response measures have also reflected that the government, enterprises, and the media are inadequate in communication. The work finally tries to provide some suggestions for solving cognitive differences, eliminating misunderstandings, and improving China's image through analyzing specific cases.

## 2. Cognitive Attitude Research Methods in the Context of Big Data

### 2.1. Big Data Algorithm Analysis

In a general analysis, the limitations of a single evaluation make the calculation result not ideal because the distribution characteristics of the processed data set are unknown. Usually, there is only one function that guides the result or the evaluation function of the result. The process is a single-objective optimization, and the result obtained often depends on an evaluation index [11]. Its distribution characteristics are not known in advance, so the evaluation mechanism for data processing should not be determined, and the applicability of the algorithm is not high. The intra-class distance and the inter-class distance of each cluster can be considered as the evaluation mechanism of clustering. Therefore, t a new evaluation function of the big-data algorithm is introduced to guide the process of clustering analysis (see Equation (1)).

(1) $$\begin{array}{c} y\left(kT+t_{i}\right)=\frac{1}{\alpha \left(z\right)}\sum_{j=1}^{r}\beta_{ij}\left(z\right)\bar{u}\left(kT+t_{j-1}\right)+v\left(kT+t_{i}\right). \end{array}$$

It can be transformed into

(2) $$\begin{array}{c} \alpha \left(z\right)=1+\alpha_{1}z^{-1}+\alpha_{2}z^{-2}+\cdots +\alpha_{n}z^{-n},\\ \beta_{ij}\left(z\right)=\beta_{ij}^{0}+\beta_{ij}^{1}z^{-1}+\beta_{ij}^{2}z^{-2}+\cdots +\beta_{ij}^{n}z^{-n}. \end{array}$$

Its function is to move sampling signal *s*(*kT*+*t*_*i*−1_)*i*=1,2,…, *r* − 1 in time backward by 1 non-uniform sampling interval *s*(*kT*+*t*_*i*−1_), and a new transfer function model is expressed as

(3) $$\begin{array}{c} y\left(kT+t_{t}\right)=\frac{B_{i}\left(\delta \right)}{A_{i}\left(\delta \right)}\bar{u}\left(kT+t_{i}\right)+v\left(kT+t_{i}\right),\\ F\left(u\right)=\int \left|Du\right|\text{d}x\text{d}y+\frac{1}{2}\lambda {\left\|u-u_{0}\right\|}^{2}. \end{array}$$

The corresponding equation is

(4) $$\begin{array}{c} -\text{div}\left(\frac{\nabla u}{\left|\nabla u\right|}\right)-\lambda \left(u_{0}-u\right)=0. \end{array}$$

For an optimization problem that can be transformed into a function, let the error function be

(5) $$\begin{array}{c} E\left(x,y\right)=\text{div}\left(\frac{\nabla u}{\left|\nabla u\right|}\right)-\lambda \left(u-u_{0}\right). \end{array}$$

Assuming that the final output is an ideal model, we can obtain

(6) $$\begin{array}{c} u\left(x,y\right)=N\left(u_{0}\left(x,y\right),w\right),\\ \frac{\text{d}I}{\text{d}s}=T\left(s\right)*\rho \left(s\right)*A=T\left(s\right)*\kappa \left(s\right). \end{array}$$

The output is

(7) $$\begin{array}{c} T=f\left(\sum_{i=1}^{n}w_{i}x_{i}-\delta \right), \end{array}$$

where *δ* represents the threshold, assuming that there are *q* pairs of samples. For the *p*th sample, the error is defined as

(8) JW,b=p12yn−y2.

where *W* represents all connection weights; *b* all connection weights in the figure; *yn* the output of the nth layer, that is, the predicted value of the entire network for the sample; *y* the true value of the sample. Calculate the average loss for the entire sample set, and then perform a uniform gradient descent.

(9) $$\begin{array}{c} J\left(W,b\right)=\frac{1}{q}\sum_{p=1}^{q}J\left(W,b\right). \end{array}$$

Find the partial derivatives and their respective contributions to the final error. This process can be expressed as

(10) $$\begin{array}{c} w_{ij}^{\left(l\right)}=w_{ij}^{\left(l\right)}-lr\frac{\partial \left(j\left(W,b\right)\right)}{\partial w_{ij}^{\left(l\right)}},\\ lr=\sigma {\left(t\right)}^{2}=w_{1}\left(t\right)*w_{2}\left(t\right)*\left(u_{1}\left(t\right)\right)-u_{1}{\left(t\right)}^{2}. \end{array}$$

where t is the threshold; *f* (*x*) the fitness function; *w*_1_(*t*) the number of nodes less than the threshold; *w*_2_(*t*) the number of nodes greater than the threshold. Generate a random number in the interval, and select the individual corresponding to the area where the random number belongs.

### 2.2. International Mainstream Media Perception

At present, there are not many influential related works that combine the fields of communication and international relations, especially the phenomenon of news communication with the theory of international relations is still lacking [12]. However, the power theory, the theory of interest, and the theory of ideology in the theory of international relations can all be used to explain the cognitive biases in journalism and communication, and the cognition and audience theory of journalism can also interpret state relations in turn. Reasons for constant conflicts [13].

At present, there are relatively few studies combining the cognition of British and American media with diplomatic behaviors. Combining media cognition with specific diplomatic events from the perspective of water protection can still improve the micro-level research of British and American media. It helps us better understand the difference between ourselves and others, and it will have a positive significance for adjusting national foreign policies and establishing multilateral cooperative relations between countries [14].

Many factors cause cognitive differences and misunderstandings in international society. In addition to national interests and the choice of diplomatic strategic objectives, specific diplomatic behaviors and diplomatic models, historical factors, cultural factors, differences in ideology and values between countries, etc. The aspect also plays an influential role that cannot be ignored [15]. In the process of diplomatic decision-making, the decision-making environment, cognitive process, and domestic factors are closely related to each other. The formulation of diplomatic decision-making is also the feedback of other influencing factors. In this process, different perceptions are likely to be formed. Even cognitive errors are due to the lack of knowledge and understanding of specific diplomatic issues and the influence of factors such as domestic culture and ideology.

The mainstream British and American media are the defenders of the interests of Western countries. Whether it is internal or external communication, the primary purpose of the British and American mainstream media is to protect their national interests. The news principle of objective reporting is always lower than the national interest. Therefore, seeking advantages and avoiding disadvantages has become a communication feature of British and American politics [16]. The mainstream British and American media are supporters of hegemonic politics. The developed countries of Britain and the United States will make full use of the power of the media to maintain their dominant position in international politics and establish a favorable international order. The main British and American media helped shape the country's image. In international political communication, the media builds the national image of other countries through the policies and events of other countries. The public cannot gain a thorough understanding of each event due to the influence of time and space. They generally learn about other countries through reports from the news media, especially mainstream media to form the image of other countries [17].

When the country conducts international political communication, it will strengthen the positive information as much as possible and weaken the negative information. Therefore, the public can establish a good national image by receiving positive information [18]. The mainstream British and American media also play the role of disseminators of the values of the British and American countries. In international politics, mainstream British and American media need to vigorously spread British and American values and mainstream ideologies, promote the political and economic systems and lifestyles of Western capitalism, gain recognition from other countries, especially socialist countries, and gain support from other countries. According to the study of media communication mode, the contents of media reports can directly or indirectly affect the audience's perception [19]. The work sorted out and analyzed the specific report texts in mainstream media in Britain and the United States and summarized the characteristics and rules. Only by recognizing the root causes of differences can we better resolve misunderstandings and conflicts in international relations.

Media have individual characteristics and can be used as the subject of “cognition” research. Different media in different countries have different cognitions and understandings of the objective world, and therefore will produce different behaviors [20]. The British and American media rely on international influence and economic power to dominate the global media landscape. The development of information technology has promoted the globalization of the media. At the same time, in the process of media globalization, the British and American media have become more and more influential in the development of international politics and international relations. They are also playing an increasingly important role in international relations [21].

We need to examine the negative side of mainstream media news websites in Britain and the United States dialectically. During the reporting period of the new crown pneumonia epidemic, British and American news websites label the virus infected by this “new crown pneumonia” as “Chinapneumonia”, “ChinaVirus”, and “Chinesecoronavirus/Chinacoronavirus”. It is not difficult to see that the various political prejudices and stereotyped inertial thinking that exist in Western society against China are accumulated and difficult to return, and the clumsy tricks of demonizing and stigmatizing China are still hard to change (see Figures 1 and 2).

There are also a lot of stigmas and false news about the epidemic in China. CNN reported the SARS epidemic in China on January 9, 2020. The United States confirmed its first epidemic and preventive measures on January 21. The number of reports began to increase rapidly, and the development of related vaccines was announced on the same day. Since late January, newspapers have often reported the closure of Wuhan, lack of medical supplies in Wuhan, WHO assessments, China's anti-epidemic measures, the withdrawal of diplomats and citizens from the United States, and social pressure. The US government is responding to the virus epidemic. On January 31, the media began to criticize the issue of racial discrimination caused by the new pneumonia epidemic. As of February 4, cases have been reported in the Hong Kong Special Administrative Region of China and the Asia-Pacific region.

Compared with other foreign media, Russia's domestic attention to the new epidemic of coronary pneumonia appeared earlier and responded more quickly. Official media such as the Russian news agency TASS and RIA Novosti paid close attention to the situation and development of the epidemic promptly and continued to pay attention. The Russian news agency TASS (TASS) reported on January 10, 2020: “According to Chinese researchers, preliminary results of laboratory tests indicate that the pathogen is a new type of coronavirus.” According to reports, the Municipal Health Commission announced the death of the first “viral pneumonia of unknown cause” in Wuhan, on January 11.

### 2.3. National Image

The “national image” has a certain degree of complexity [22]. To put it simply, “national image” can be divided into “self-image” and “other-view image”. According to the different cognitive subjects and nature, its manifestation also has certain differences. From the point of view of the cognitive subject, if the cognitive subject is the people of the country, this is a kind of domestic image, which is the so-called “self-image”. If the cognitive subject is transformed into the government or the people of another country, it will become the so-called “other-view image”.

In Figure 3, according to the Pew Research Center's 2015 spring US global public opinion survey, we can see the evaluation of various countries on China, and the countries that have a good impression of China are mainly concentrated in Africa, Latin America, etc.[23].

Strictly speaking, the issue of China's image studied in this article, that is, the issue of “other-view image”, should be classified as an issue of international image rather than a broad category of national image. The international image of a country is very different from the national image of this country. “There can be complete divergence, a long distance, roughly the same, infinite closeness, complete unity (this kind of situation is unlikely), etc. between the two. Circumstances.” Some international statements about “China's demonization” have further deepened the importance of distinguishing between the international image and the national image. “The international image of a country is the comprehensive cognition and evaluation of a country's political, economic, social, cultural, diplomatic and natural elements by the international community.” “The international image of a country is mainly manifested as a diplomatic image and its status among the international public. So the work mainly started from one of the manifestations of the international image, the international media, and subdivides reports on Chinese tourists from the report content and used them as a starting point to analyze the issue of China's international image [24].

The discourse of the international community has always been in the hands of developed countries such as the United Kingdom and the United States for a long time. National interests are the fundamental factor influencing national policy choices. The lack of media discourse power has caused many of China's diplomatic behaviors to be misinterpreted by the British and American media, which interferes with the public's perception. This project hopes to take the aid to Africa incident as the starting point, call China and other developing countries to attach importance to their national image, understand the understanding of the British and American mainstream media on their country's diplomatic behavior, and develop the domestic media's international visibility and credibility. The original truth of the matter will better promote China's foreign affairs with other related countries.

The media play a key role in shaping and disseminating a country's international image. As the media of different countries maintain different values and represent different interests, there will be some differences in the social phenomena that are reflected. It is believed that even within a country, the phenomena reported by different media will be inconsistent with each other [25]. Therefore, the work selected two media with different tendencies for further research.

## 3. Experiment on Mainstream Media's Perception and Attitude Towards China

### 3.1. Research Samples

All the news data in the work come from LexisNexisAcademicUniverse, a sub-database of Databases@Emory of Emory University. We used “China (China)” and “Covid-19” as keywords, and selected the period from December 1, 2019, to April 31, 2021. We received relevant news and analyzed the content of their reports. After the screening, valid reports were retained (including 135 in The New York Times, 125 in The Times, and 109 in the Guardian). The main content of the report includes the number of people infected with water pollution in China, pollution source virus, national reviews, etc.

### 3.2. Establishing a Model Evaluation Index System

A clear conclusion can be drawn through actual observation of the object. Generally speaking, the evaluation index system includes three levels of evaluation indexes: they are the relationship between gradual decomposition and refinement. The first-level evaluation indicators and the second-level evaluation indicators are relatively abstract and cannot be used as a direct basis for evaluation. The third-level evaluation indicators should be specific, measurable, and behavior-oriented, and can be used as a direct basis for teaching evaluation.

### 3.3. Determine the Evaluation Weight

The index weight is a numerical index indicating the importance and function of the index. In the indicator system of the evaluation plan, the weight of each indicator is different. Even if the indicator level is the same, the weight is different. Index weight is also called weight and is usually represented by a. It is a number greater than zero but less than 1, and the sum of the weights of all first-level indicators must be equal to 1, that is, satisfy conditions 0 < *a* < 1 and ∑a-1.

### 3.4. Statistics

All data analysis in the work used SPSS19.0, and the statistical test used a two-sided test. Significance was defined as 0.05, and *p* < 0.05 was considered significant. The statistical results were displayed as mean ± standard deviation (*x* ± SD). When the test data obeyed the normal distribution, the double *T*-test was used for comparison within the group, and the independent sample *T*-test was used for comparison between the groups. If the regular distribution was not sufficient, two independent samples and two related samples were used for inspection.

## 4. Experimental Analysis of Mainstream Media's Cognitive Attitude Towards China

### 4.1. Mainstream Media Reports

We first made relevant statistics on the reports of the international mainstream media on China during water pollution and compared the differences in reports between different media (see Table 1).

Table 1 shows that media reports on China are extremely frequent, and every report is designed during water pollution. The propaganda and media systems of various countries in the world can be roughly divided into four theoretical types, namely, authoritarian theory, liberal theory, social responsibility theory, and communist (total) theory type.” China uses the communism theory, while Japan uses it. This is the theoretical basis of liberalism. They have their unique views on the attitude of their governments due to the different processes of the historical development of the big newspapers.

The distribution of the number of reports on China in the water pollution over time by the New York Times, The Times, and the Guardian since the outbreak of the water pollution (see Table 2).

Table 2 shows that the name of the report has been changed many times before and after, using “Water Pollution” 380 times, “Domestic Wastewater” 12 times, “Industrial Wastewater” 12 times, and “Industrial Wastewater” 8 and 3 times, “Agricultural Wastewater” 3 times, “Industrial Wastewater” 5 times, “Agricultural Wastewater” 1 time, and “Town Wastewater” 1 time.

Immediately after the epidemic broke out in China (See Table 3), we calculated the number of reports from these media and the number of positive and negative reports based on time points. (See Figure 4).

When water pollution first appeared in China, foreign media began to pay attention to it, and the relevant articles gradually increased, with overall positive and negative references. The international media's overall coverage of the water pollution in China has been ideologically in command, full of these colored glasses. Especially when Wuhan was closed on January 3, 2020, mainstream media in Europe and the United States showed negative reports. It is authoritarianism to criticize China for infringing on people. Of course, internationally, there are related media expressing support for China's measures.

### 4.2. Length of Media Coverage

The length of a related report is the number of words in each related report. Generally speaking, the larger the length of a report, the greater its influence and the stronger the desire for the relevant content to be conveyed. In the statistical process of the length of relevant reports, they are divided into newsletters, news, reports, and in-depth reports according to the law of communication. We have made statistics on the length of these reports (see Figure 5).

Judging from the overall report, the number of words in the report is 4,258, and that of words is 86. There are 161 articles with a length of fewer than 200 words, accounting for 43.6% of the total; 85 articles with more than 200 and less than 800 words, accounting for 23% of the total; 79 articles with a length of more than 800 and less than 2,000 words, accounting for 21.4% of the total. There are 44 articles with more than 2000 words, accounting for 12% of the total. Among these reports, the related negative reports mainly involve “human rights issues”, “corruption and autocracy”, “man-made viruses”, “virus experiments”, etc (see Figure 6).

In the overall report, the main reports of these three media still show a trend of negative reports. They repeatedly criticized water pollution prevention measures for infringing human rights and being an authoritarian country. Of course, some of the readers of these media were persuaded by the media's remarks, but some were dissatisfied with the contaminated source virus treatment in foreign countries, hoping that they would learn from China's virus treatment control and protect the people's health of the country (see Figure 7 for the details).

In the comments of the reader, more and more readers have questioned the objectivity of the “New York Times” report, believing that this analysis has many subjective problems and is entirely propaganda for the Western government. There is no doubt that the ownership of the media and the control of national political power has a major impact on the shaping of the international political news framework.

## 5. Conclusions

The Chinese and British and American media coverage of the same event will inevitably be influenced by their respective cultural forms due to differences in cultural values, which creates significant differences between Chinese and British and American media reports and forms significant differences between Chinese and British and American media reports. From the reporting standpoint, the mainstream media in Britain and the United States still have a clear Cold War color. Starting from the ideological and cultural background, they choose and determine the tendency of news reporting. The ultimate goal is to include China in the United Kingdom and the United States and realize the unanimity of the ideology of the international community as the leading international system.

Chinese media should change the current political propaganda orientation, adhere to the principle of objectivity, and return news reports to the incident. It should report on achievements and face up to the existing problems and the views and attitudes of other countries. Domestic media should increase the transparency of information from the source to ensure the authenticity, objectivity, and efficiency of news reports and avoid the tendency of Western media reports.

## Figures and Tables

**Figure 1:** BBC's return to Wuhan's China-related report “Underworld Filter”. (a) BBC Chinese Report. (b) BBC English report.

**Figure 2:** The New York Times reported that China and Italy were closed when cities were closed. (a) The New York Times reported when the city was closed in China. (b) The New York Times reported when the city was closed in Italy.

**Figure 3:** Senses of other countries and regions to China.

**Figure 4:** Number of positive and negative reports.

**Figure 5:** Report length.

**Figure 6:** Topic popularity.

**Figure 7:** Readers' comments.

**Table 1:** Number of reports by different media.

Numbering	Media	Country	Number of reports
1	New York Times	United States	941
2	Times	United Kingdom	662
3	Guardian	United Kingdom	413
4	Asahi Shimbun	Japan	381
5	USA Today	United States	330
6	Awakening Daily	India	316
7	Daily news	Japan	307
8	Times of India	India	293
9	Nihon Keizai Shimbun	Japan	27

**Table 2:** Media coverage of water pollution.

	China	Water pollution	Domestic Wastewater	Industrial Wastewater	Agricultural Wastewater	Town Wastewater
New York Times	253	152	132	8	3	1
Times	235	132	117	3	1	0
Guardian	185	155	131	1	1	0

**Table 3:** The amount of information released by the media over time.

	December 26, 2019	December 31, 2019	January 3, 2020	January 23, 2020	March 10, 2020
New York Times	8	11	25	33	17
Times	5	10	12	36	12
Guardian	4	8	12	32	10

## Data Availability

The data used to support the findings of the work are available from the corresponding author upon request.
